The article "Gene Differential Expression and Interaction Networks Illustrate the Biomarkers and Molecular Mechanisms of Atherosclerotic Cerebral Infarction" was published in 2022. Journal: J Healthc Eng.

# Gene Differential Expression and Interaction Networks Illustrate the Biomarkers and Molecular Mechanisms of Atherosclerotic Cerebral Infarction

**DOI:** 10.1155/2022/3912697

**Published:** 2022-01-12

**Authors:** Benzhuo Zhang, Wei Huang, Mingquan Yi, Chunxu Xing

**Affiliations:** ^1^Department of Neurology, The Second Affiliated Hospital of Mudanjiang Medical College, Mudanjiang 157000, Heilongjiang, China; ^2^Academic Affair Office, Mudanjiang Medical University, Mudanjiang 157011, Heilongjiang, China; ^3^Medical Department of the Second Affiliated Hospital of Mudanjiang Medical College, Mudanjiang 157000, Heilongjiang, China; ^4^Department of Traditional Chinese Medicine, The Second Affiliated Hospital of Mudanjiang Medical College, Mudanjiang 157000, Heilongjiang, China

## Abstract

Atherosclerotic cerebral infarction (ACI) seriously threatens the health of the senile patients, and the strategies are urgent for the diagnosis and treatment of ACI. This study investigated the mRNA profiling of the patients with ischemic stroke and atherosclerosis via excavating the datasets in the GEO database and attempted to reveal the biomarkers and molecular mechanism of ACI. In this study, GES16561 and GES100927 were obtained from Gene Expression Omnibus (GEO) database, and the related differentially expressed genes (DEGs) were analyzed with R language. Furthermore, the DEGs were analyzed with Gene Ontology (GO) and Kyoto Encyclopedia of Genes and Genomes (KEGG) enrichment analysis. Besides, the protein-protein interaction (PPI) network of DEGs was analyzed by STRING database and Cytoscape. The results showed that 133 downregulated DEGs and 234 upregulated DEGs were found in GES16561, 25 downregulated DEGs and 104 upregulated DEGs were found in GSE100927, and 6 common genes were found in GES16561 and GES100927. GO enrichment analysis showed that the functional models of the common genes were involved in neutrophil activation, neutrophil degranulation, neutrophil activation, and immune response. KEGG enrichment analysis showed that the DEGs in both GSE100927 and GSE16561 were connected with the pathways including Cell adhesion molecules (CAMs), Cytokine-cytokine receptor interaction, Phagosome, Antigen processing and presentation, and *Staphylococcus aureus* infection. The PPI network analysis showed that 9 common DEGs were found in GSE100927 and GSE16561, and a cluster with 6 nodes and 12 edges was also identified by PPI network analysis. In conclusion, this study suggested that FCGR3A and MAPK pathways were connected with ACI.

## 1. Introduction

Cerebral infarction is the second fatal disease in modern society, which is a global issue threatening the health of humans. Statistically, more than 70% cerebral infarction is induced by ischemia, and ACI serves as a major type in it [1, 2]. Atherosclerotic cerebral infarction (ACI) is a complex disease in clinical. Atherosclerosis has been confirmed as a major reason leading to the progression of ischemic stroke [3, 4]. For atherosclerosis, imaging diagnostic technologies have been widely applied for early warning of symptoms, and the intervention of drugs and surgeries on vessel could also effectively improve the symptom of the patients [5]. Many studies have indicated that accumulated lipids and foam cells are main reasons for ACI development. However, the known proofs are still far from the fully clear molecular mechanism of ACI [6]. Moreover, even with current medical technologies, the diagnostic and therapeutic effects on ACI remain unsatisfactory [7, 8]. Therefore, more biomarkers and deep molecular mechanism are necessary for ACI treatment.

The article "Gene Differential Expression and Interaction Networks Illustrate the Biomarkers and Molecular Mechanisms of Atherosclerotic Cerebral Infarction" was published in 2022. Journal: J Healthc Eng.

High-throughput screen is characterized with high efficiency and accuracy in gene sequencing, which has been increasingly applied in clinical research [9]. Microarray analysis has also been widely applied to illustrate the molecular mechanisms and diagnostic biomarkers in various diseases, which effectively promote the development of the researches in multiple diseases [10]. The proofs have revealed the difference in gene profiling of the patients and the normal persons, and some factors play important roles in the formation and development of ischemic stroke [11]. Moreover, increasing studies have identified the differentially expressed genes as the biomarkers in the patients with ischemic stroke. For instance, Gu et al. have identified the therapeutic targets for atherosclerosis by analyzing GSE107522 [12].

Therefore, this study attempted to identify the differentially expressed genes (DEGs) of the patients and normal persons and investigate the pathological mechanism of ischemic cerebral infarction induced by atherosclerosis by delving the microarray datasets in Gene Expression Omnibus (GEO) database.

## 2. Materials and Methods

### 2.1. Data Acquisition

The microarray datasets including GES16561 and GES100927 were obtained from National Center Biotechnology Information Gene Expression Omnibus (https://www.ncbi.nlm.nih.gov/geo/). The samples of 39 patients with stroke and 24 normal individuals in GES16561 tested on GPL6883 were selected for subsequent analysis, and the samples of 29 patients with carotid atherosclerosis and 24 normal persons in GSE100927 were selected for subsequent analysis.

### 2.2. Identification of Differentially Expressed Genes

The datasets were analyzed with the limma package by R language with a moderate t-test corrected by Benjamini and Hochberg's methods (adjusted p value <0.05. Moreover, the genes with the Log fold change (log FC) > 2 were selected as DEGs.

The article "Gene Differential Expression and Interaction Networks Illustrate the Biomarkers and Molecular Mechanisms of Atherosclerotic Cerebral Infarction" was published in 2022. Journal: J Healthc Eng.

### 2.3. Gene Function and Pathway Analysis

The Gene Ontology analysis was performed to identify the functions of the DEGs in GSE16561 and GSE100927. In brief, the packages including clusterProfiler and topGO were preloaded in R studio, and the ENTREZIDs of the DEGs obtained from DAVID(https://david.ncifcrf.gov/) were analyzed to reveal the functions of the DEGs. After that, the results were visualized by topGO package. The Kyoto Encyclopedia of Genes and Genomes (KEGG) were performed on DAVID and then the results were visualized with ggplot2 package.

### 2.4. Protein-Protein Interaction (PPI) Network Analysis

The interaction of the DEGs was performed by protein-protein interaction network (PPI) analysis. In brief, the DEGs of datasets were uploaded on STRING database (http://string-db.org) to obtain the results of PPI network, and then the results were further analyzed with Cytoscape (version 3.7.1).

## 3. Results

### 3.1. Identification of Differentially Expressed Genes

To reveal the profiling difference of genes in the patients and normal persons, the clinical microarray datasets including GES16561 and GES100927 were analyzed by limma package. The results showed that 134 downregulated DEGs and 234 upregulated DEGs were found in GES16561 and 25 downregulated DEGs and 104 upregulated DEGs were found in GSE100927 (Figures 1 and 2). Moreover, it was found that 9 common genes were found in GES16561 and GES100927 including AQP9, CD2, FCGR3A, ITGAM, MMP9, and NPL (Figure 1(c)).

### 3.2. Gene Function Analysis

To delve the molecular functions of DEGs, the GO enrichment analysis was performed. The results showed that the DEGs in GSE16561 were enriched into 100 related molecular functions, and the DEGS in GSE100927 were enriched into 268 molecular functions. Moreover, for GSE16561, the DEGs were involved in neutrophil activation, neutrophil degranulation, neutrophil activation involved in immune response, neutrophil-mediated immunity, and so on (Figure 3). For GSE100927, the DEGs were also related to neutrophil activation, neutrophil degranulation, and neutrophil activation involved in immune response (Figure 3).

### 3.3. Gene Pathway Analysis

To explore the regulation mechanism of DEGs, the DEGs of GSE16561 and GSE100927 were analyzed by KEGG enrichment analysis. The result have indicated that 68 DEGs in GSE100927 were enriched in 18 pathways and 163 DEGs in GSE16561 were enriched in 16 pathways. For GSE100927, the DEGs were involved in *Staphylococcus aureus* infection, Osteoclast differentiation, Leishmaniasis, Chemokine signaling pathway, Phagosome, and so on. For GSE16561, the DEGs were involved in Primary immunodeficiency, Hematopoietic cell lineage, T cell receptor signaling pathway, *Staphylococcus aureus* infection, Tuberculosis, and so on (Figure 4). Moreover, some DEGs in both GSE100927 and GSE16561 were connected with the pathways including Cell adhesion molecules (CAMs), Cytokine-cytokine receptor interaction, Phagosome, Antigen processing and presentation, and *Staphylococcus aureus* infection (Figure 4).

The article "Gene Differential Expression and Interaction Networks Illustrate the Biomarkers and Molecular Mechanisms of Atherosclerotic Cerebral Infarction" was published in 2022. Journal: J Healthc Eng.

### 3.4. Protein-Protein Network Analysis

To further reveal the molecular mechanism of the genes in the progression of ischemic stroke induced by atherosclerosis, the interactions of DEGs were analyzed by STRING database and Cytoscape. According to the MCODE analysis, the clusters of the top three scores of GSE100927 and GSE16561 were selected for visualization. For GSE16561, cluster 1 involved 23 nodes and 348 edges, cluster 2 involved 19 nodes and 158 edges, and cluster 3 involved 8 nodes and 40 edges (Figures 5(a)–5(c)). For GSE100927, cluster 1 involved 16 nodes and 196 edges, cluster 2 involved 5 nodes and 20 edges, and cluster 3 involved 6 nodes and 20 edges (Figures 5(d)–5(f)). Besides, 6 common DEGs were found in GSE100927 and GSE16561, and a cluster with 6 nodes and 12 edges was also identified by PPI network analysis (Figure 5(g)).

## 4. Discussion

Increasing studies have indicated that the development of cerebral infarction induced by atherosclerosis is one of the major types of ischemic stroke [13]. Although the pathogenic mechanism of ACI has been increasingly revealed, more biomarkers are urgent for diagnosis and treatment. In this study, the clinical datasets were obtained from NCBI and used to analyze the difference of the expressed genes in the patients and normal individuals, GO and KEGG enrichment analyses were performed to further investigate the functions and related pathways of the DEGs, and PPI network analysis was used to reveal the molecular mechanism of the potential factors.

Atherosclerosis has been thought as the major reason of ischemic stroke [14]. Plaque rupture may induce the carotid arterial embolism and finally causes acute ischemic stroke. Guo et al. have indicated that the diagnostic results of atherosclerosis could provide effective guidelines for the patients with ischemic stroke [15]. In this study, GSE16561 including the samples of the patients with stroke and GSE100927 including the samples of the patients with atherosclerosis were analyzed. It was found that the patients with atherosclerosis or ischemic stroke exhibited significant difference in gene profiling and 9 common genes were found in GES16561 and GES100927 including AQP9, CD2, CD3D, CD8A, FCGR3A, ITGAM, KCNJ15, MMP9, and NPL, suggesting that the DEGs were related to the progression of ACI.

The article "Gene Differential Expression and Interaction Networks Illustrate the Biomarkers and Molecular Mechanisms of Atherosclerotic Cerebral Infarction" was published in 2022. Journal: J Healthc Eng.

The progression of ACI is related to the abnormal expression of multiple genes. In this study, the DEGs of GSE16561 and GSE100927 were analyzed by GO enrichment analysis. It was found that the DEGs in GSE16561 and GSE100927 were also related to neutrophil activation, neutrophil degranulation, and neutrophil activation involved in immune response, which suggests that both atherosclerosis and ischemic stroke are connected with the abnormally activation of the neutrophils. Neutrophils involve the various inflammatory reactions, and the inflammation induced by neutrophils has been confirmed to play the major roles in the formation of atherosclerosis [16]. The study has indicated that neutrophils can interact with the platelets to mediate the activation of TLR4/NF-*κ*B pathway [17]. Denorme et al. have also indicated that platelet-neutrophil interaction could also aggravate ischemic stroke [18]. Moreover, it was also found that both atherosclerosis and ischemic stroke were related to cellular adhesion and leukocyte cell-cell adhesion. The disorder in cellular adhesion promotes cell aggregation and then boosts the formation of plaques, and accumulating proofs have supported that large clusters of cells are the main reason causing plaque rupture. Increased vascular cell adhesion molecules have also been found in the patients with atherosclerosis [19]. The study of Wei et al. has also indicated that platelet-endothelial cell adhesion molecule-1 is also related to ischemic stroke [20]. Besides, this study also found that the DEGs of GSE16561 and GSE100927 were associated with the regulation of immune effector process. Cardiovascular inflammation and disturbed interactions between circulating immune cells and the vascular system are key drivers of atherosclerosis, and some key immune factors have been thought as the promising therapeutic target of atherosclerosis [21, 22]. Thus, those proofs suggest that neutrophil activation, cellular adhesion, and the regulation of immune effector process are involved in the progression of ACI.

This study confirmed that the DEGs in GSE16561 were enriched in Herpes simplex infection, Viral carcinogenesis, Cytokine-cytokine receptor interaction, MAPK signaling pathway, and HTLV-I infection pathways, while the DEGs in GSE100927 were enriched in Phagosome, Transcriptional misregulation in cancer, Tuberculosis, Chemokine signaling pathway, and Cytokine-cytokine receptor interaction pathways. However, it was also found that both GSE16561 and GSE100927 were enriched in MAPK, Cytokine-cytokine receptor interaction, antigen processing and presentation, and cGMP-PKG signaling pathways. MAPK pathway is implicated in various cellular activities including cell apoptosis and inflammation [23, 24]. Abnormally activated MAPK pathways serve as a major role in the development of multiple inflammations, and targeting MAPK pathways have been proved to effectively alleviate the symptom of atherosclerosis [25]. Besides, inhibited MAPK pathway could also significantly improve the cognitive impairment induced by ischemic stroke [26]. Thus, this study supports that aberrant activation of MAPK pathway takes a great part in the progression of atherosclerotic cerebral infarction.

The article "Gene Differential Expression and Interaction Networks Illustrate the Biomarkers and Molecular Mechanisms of Atherosclerotic Cerebral Infarction" was published in 2022. Journal: J Healthc Eng.

PPI network analysis has been confirmed as an effective strategy for tracking genes and investigating molecular mechanism of diseases [27]. In this study, PPI network analysis was also used to reveal the regulation mechanism of the DEGs. For GSE16561, CD8A, ITGAM, FCGR3A, CD19, CD2, HIF1A, and CREBBP acted as the key nodes in DEGs, and ITGAM, FCGR3A, MMP9, and CD68 served the key roles in DEGs of GSE100927. Furthermore, it was found that FCGR3A was the key nodes in 6 common genes of GSE16561 and GSE100927. FCGR3A is also named as CD16 which has been identified as the pathogenic factor to participate in the deterioration of atherosclerosis, and the study has indicated that FCGR3A may be connected with ischemic stroke [12, 28]. Besides, several studies have shown that both FCGR3A and MAPK pathway exhibited significant aberrant levels in some diseases such as chronic constriction and Periodontitis [29, 30], while few studies have indicated the connection of FCGR3A and MAPK pathway.

## Figures and Tables

**Figure 1:** Volcano plots of differentially expressed genes between patients with ACI and related controls. Red nodes denote upregulation and blue nodes denote downregulation. (a) The expressed genes of GSE16561. (b) The expressed genes of GSE100927. (c) The common genes of GSE16561 and GSE100927 exhibited by Venn diagram.

**Figure 2:** Heat maps of differentially expressed genes between patients and related controls. (a) GSE16561. (b) GSE16561. Orange represents upregulation and blue represents downregulation.

**Figure 3:** The modular functions involved in ACI development. (a). Module gene GO enrichment analysis of GSE16561. (b) Module gene GO enrichment analysis of GSE100927.

**Figure 4:** The pathways involved in ACI development. (a) Module gene KEGG enrichment analysis of GSE16561. (b) Module gene KEGG enrichment analysis of GSE100927. The larger the size, the more significant the proportion of the gene.

**Figure 5:** The PPI network of DEGs in ACI. (a–c) The PPI network of GSE16561. (d–f) The PPI network of GSE100927. (g) The PPI network of common genes.

The article "Gene Differential Expression and Interaction Networks Illustrate the Biomarkers and Molecular Mechanisms of Atherosclerotic Cerebral Infarction" was published in 2022. Journal: J Healthc Eng.

## Data Availability

Data used to support the findings of this study are available from the corresponding author upon reasonable request.
